The article "Clinical and Laboratory Biomarkers in Paroxysmal Atrial Fibrillation: A Single Center Cross-Sectional Study" was published in 2022. Journal: Contrast Media Mol Imaging.

# Clinical and Laboratory Biomarkers in Paroxysmal Atrial Fibrillation: A Single Center Cross-Sectional Study

**DOI:** 10.1155/2022/7012377

**Published:** 2022-06-29

**Authors:** Weiping Sun, Haiwei Li, Zefeng Wang, Yongquan Wu, Jia Du

**Affiliations:** ^1^Beijing Institute of Heart, Lung and Blood Vessel Disease, Beijing Anzhen Hospital, Capital Medical University, Beijing, China; ^2^Department of Cardiology, Beijing Anzhen Hospital, Capital Medical University, Beijing, China

## Abstract

The clinical risk profile of paroxysmal atrial fibrillation (pAF) patients is inconclusive. We aimed to identify clinical and laboratory biomarkers in patients with pAF and the differences in biomarkers among genders. A cross-sectional study was conducted with a total of 181 participants in a single center in Beijing Anzhen Hospital. The participants were grouped according to the presence of pAF and sex differences, and clinical and laboratory results were collected and compared. The 181 participants had a mean age of 52.9 ± 15.1 years (pAF group, 60.4 ± 9.9 years, SR group, 48.3 ± 15.9 years, *P* < 0.05). Patients with pAF had significantly higher rates of age, left atrial (LA) diameter, haemoglobin (Hb) levels, tissue inhibitor of metalloproteinase-1 (TIMP-1), soluble tumour suppressor-2 (sST2), B-type natriuretic peptide (BNP) and indirect bilirubin (Ibil), mean haemoglobin concentration (MCHC), and hypertension (HTN) and smoking (*P* < 0.05). Multivariable logistic regression analysis revealed that age (OR = 1.075, 95% CI: 1.035–1.118, *P* < 0.0001), smoking (OR = 4.538, 95% CI: 1.559–13.205, *P* = 0.006), and MCHC (OR = 1.062, 95% CI: 1.019–1.106, *P* = 0.004) were independent predictive factors for pAF. Multivariable logistic regression analysis found that age (OR = 1.107, 95% CI: 1.016–1.206, *P* = 0.02) and Ibil level (OR = 2.303, 95% CI: 1.158–4.582, *P* = 0.017) were independent predictive factors of the occurrence of pAF in females; BNP (OR = 1.015, 95% CI: 1.002–1.029, *P* = 0.029) was an independent predictive variable of pAF in males. Age, smoking, and MCHC were independent predictive factors of pAF. BNP was an independent predictive biomarker of pAF in males, while in females, age and Ibil were independent predictive factors.

## 1. Introduction

Atrial fibrillation (AF) is the most common sustained arrhythmia encountered in clinical practice [1]. AF is associated with substantial morbidity and mortality, therefore leading to a significant burden on patients, societal health, and economic development [2]. The prevalence of atrial fibrillation in adults is currently estimated to be between 2% and 4%, and a recent study suggests that an estimated 1 in 3 people were at risk of developing atrial fibrillation by the age of 55 [3, 4]. Paroxysmal atrial fibrillation (pAF) has a higher incidence and risk in adults. At present, the mechanism of atrial fibrillation is not fully understood; the AF lifetime risk depends on age and genetic and clinical factors [1, 5]. Early intervention and modifiable risk factor control could reduce the incidence of AF; therefore, identifying the risk factors for pAF is of great significance for the prevention of AF.

Recent studies have revealed sex-related differences in the clinical presentation, pathogenesis, outcomes, and management of AF patients; specifically, the risk of developing AF is 1.5–2.0 times higher in males than in females [6]. The cumulative AF incidence increases after the age of 50 years in males and 60 years in females; however, the lifetime risk is similar (>30%) between the sexes [3].

Regarding biomarkers for AF, guidelines for patient management have shown that serum N-terminal prohormone B-type natriuretic peptide (NT-proBNP) is a more powerful biomarker than other clinical variables, as well as echocardiographic assessment (left atrial and ventricular diameters) [2]. Recent studies have also found that soluble isoform of ST2 (sST2), tissue inhibitor matrix metalloproteinase 1 (TIMP-1), high-sensitivity C-reactive protein (hs-CRP), and BNP are involved in the mechanism of AF. Unfortunately, the precise mechanisms and signaling pathways involved in the atrial remodeling processes of AF have not been completely elucidated, and data on biomarkers as predictors of pAF are limited. Therefore, the aim of this study was to investigate potential clinical biomarkers that could be used to predict the occurrence of pAF, providing a theoretical basis for AF interventions and to identify biomarker and risk factor differences in females and males with pAF.

## 2. Methods

### 2.1. Study Design

The purposes of this cross-sectional study were to explore (i) potential clinical and laboratory biomarkers that could be used in predicting paroxysmal AF and (ii) differences in biomarkers and their values between females and males with pAF. The independent variables of this study came from clinical and laboratory examinations.

### 2.2. Participants

This study was approved by the ethics committee of Beijing Anzhen Hospital. In this cross-sectional study, 68 consecutive inpatients referred to our hospital for paroxysmal atrial fibrillation were included from June 2018 to July 2019 at the Beijing Anzhen Hospital. Simultaneously, we enrolled 113 inpatients with sinus rhythm (SR) as controls. The inclusion criteria were age greater than 18 years; clinical diagnosis with pAF; informed consent to participate in this study; and submission of a signed informed consent form. The exclusion criteria were AF or other heart diseases after inclusion in the SF group; diagnosis with persistent or permanent atrial fibrillation; presence of malignant tumors with a life expectancy shorter than 1 year; or other end-stage diseases. The definition of paroxysmal AF was AF that terminates spontaneously or with intervention within 7 days of onset; it was diagnosed based on 12-lead electrocardiogram and 24-hour ambulatory electrocardiogram.

### 2.3. Data Collection

General data of patients were collected, including age, sex, hypertension, coronary artery disease (CAD), diabetes, heart failure, and other indicators. At the same time, the clinical examination and laboratory results of the patients were collected, including white blood cell (WBC), red blood cell (RBC), platelet count (PLT), haemoglobin (Hb), fasting blood glucose, fibrinogen, D-dimer, creatinine, urea, uric acid (UA), aspartate transaminase (AST), alanine aminotransferase (ALT), lipoprotein, total cholesterol (TC), triacylglycerol (TG), and low-density lipoprotein (LDL). Left atrium (LA) diameter, left ventricular end-systolic dimension (LVESD), left ventricular end-diastolic dimension (LVEDD), and left ventricular ejection fraction (LVEF) were measured. For the blood markers, from the same blood sampling as TIMP-1, sST2, hs-CRP, and BNP, for other assessments, within 6 h of blood sampling. The CHA2DS2-VASc score and HAS-BLED score were also assessed in all participants.

### 2.4. Statistical Analysis

All statistical analyses were performed using Statistical Product and Service Solutions (SPSS) 20.0 (IBM Corp., Armonk, NY, USA). Continuous data are expressed as the mean ± standard deviation and were analyzed by Student's *t*-test (comparisons of two groups). Nonnormally distributed continuous data are described as the median and interquartile range (IQR) and were compared using the Wilcoxon rank-sum test. Categorical variables are presented as numbers (percentages) and were analyzed by the Chi-square test or Fisher's exact test, as appropriate. Parameters with *P* < 0.05 in the univariable analysis were included in the multivariable logistic regression analysis by the enter method. *P* < 0.05 was considered statistically significant.

## 3. Results

### 3.1. Baseline Clinical and Laboratory Participant Characteristics

A total of 181 participants were enrolled in our study. The 181 participants had a mean age of 52.9 ± 15.1 years (pAF group, 60.4 ± 9.9 years and SR group, 48.3 ± 15.9 years). Sixty-eight patients (46 males and 22 females) were included in the pAF group. The baseline clinical and laboratory characteristics of the participants are shown in Tables 1 and 2. Patients with pAF had significantly higher age, levels of Hb, creatinine, TIMP-1, sST2, Tbil, Ibil, and major histocompatibility complex (MHC), MCHC, and proportions of HTN and smoking (Figure 1). The levels of PLT, TP, Alb, and HDL-c in the pAF group were lower than those in the SR group.

### 3.2. Multivariable Logistic Regression Analysis of Factors Associated with pAF

Multivariable logistic regression analysis was performed in the pAF group following the univariable logistic regression analysis. The results revealed that age (OR = 1.075, 95% CI: 1.035–1.118, *P* < 0.0001), smoking (OR = 4.538, 95% CI: 1.559–13.205, *P* = 0.006), and MCHC (OR = 1.062, 95% CI: 1.019–1.106, *P* = 0.004) were independent predictive factors of pAF. Detailed results of the multivariable analysis are shown in Table 3.

### 3.3. Clinical Characteristics and Risk Factor Differences between Males and Females with pAF

As shown in Table 4, males had higher levels of Hb, CREA, TIMP-1, Tbil, Ibil, and MHC, MCHC, and proportion of smokers than females in the pAF group. Further multivariable logistic regression analysis (Table 5) showed that age (OR = 1.107, 95% CI: 1.016–1.206, *P* = 0.02) and Ibil (OR = 2.303, 95% CI: 1.158–4.582, *P* = 0.017) were independent predictive factors of the occurrence of pAF in females. BNP (OR = 1.015, 95% CI: 1.002–1.029, *P* = 0.029) was an independent predictive variable of pAF in males.

## 4. Discussion

The main findings of this study are as follows: (I) the pAF group was older and had higher levels of TIMP-1, sST2, and Ibil and a higher MCHC; moreover, smoking was more likely to be seen in the pAF group. (II) Multivariable logistic regression analysis showed that age, smoking, and MCHC were independent predictive factors of pAF. (III) Subgroup analysis based on sex showed that males with pAF had higher levels of Hb, CREA, TIMP-1, and Ibil, a higher MCHC, and a higher proportion of smokers than females; females with pAF had higher levels of PLT, UA, and HDL-c. (IV) Multivariable logistic regression analysis found that age and Ibil were independent predictive factors of the occurrence of pAF in females; BNP was an independent predictive variable of pAF in males.

Risk factors for AF progression include age, heart failure (HF), hypertension, chronic kidney disease (CKD), diabetes mellitus (DM), previous stroke, and left atrial size, but the added predictive value of biomarkers is presently not well defined [7]. Studies have revealed that older age is associated with permanent AF, but the correlation with pAF is unclear [2, 8]. In our study, we found that the pAF group was older, and multivariable analysis revealed that age was an independent predictive factor for pAF in females. Meanwhile, the pAF group also had a larger LA size, which was consistent with a previous study [7]. This reflects, to some extent, that AF was also a marker of atrial structural remodeling.

Serum ST2 is a member of the interleukin-1 receptor family, and circulating sST2 concentrations are believed to reflect cardiovascular stress and cardiac fibrosis. Receptor ST2L is involved in the inhibition of cardiac hypertrophy and fibrosis [9]. High concentrations of sST2 can prevent this protective effect and lead to cardiac fibrosis, which is linked to atrial fibrillation via arrhythmogenic structural remodeling [10]. However, the role of soluble ST2 in pAF has not been previously explored. Okar and colleagues reported that soluble ST2, as measured prior to an ablation procedure, is an independent parameter for predicting AF recurrence [11]. Other studies have suggested that sST2 was associated with LA volume enlargement, the LA low-voltage zone, and LV myocardium abnormalities in patients with paroxysmal AF [12, 13]. Similar to the above findings, our results indicate that the median sST2 concentration of the pAF group was 12.76 ± 4.73 ng/ml, higher than that of the SR group.

Atrial structural remodeling and maintenance of the extracellular space includes not only synthesis but also coordinated degradation of extracellular matrix (ECM) proteins (matrix metalloproteinases (MMPs) and TIMPs). Under normal circumstances, TIMP-1 inhibits the enzymatic activity of MMP-9 and regulates ECM turnover. However, the levels of TIMP-1 in pAF patients are not yet known. Paulina et al. found that the levels of TIMP-1 in pAF patients are elevated [14]. In contrast, another study showed that TIMP-1 serum levels were lower in paroxysmal and persistent AF [15]. In the current study, the pAF group also had elevated TIMP-1, but the reason for the difference in TIMP-1 levels was unclear. An imbalance between MMPs and TIMPs may reflect abnormal turnover of the ECM and therefore results in atrial remodeling and fibrosis.

NT-proBNP has been reported to be a predictor of AF in atrial fibrillation guidelines, but the use of baseline BNP levels as a predictor for pAF is inconclusive [2]. In the present study, the pAF group had a higher level of BNP than the SR group, and further multivariable analysis showed that BNP was an independent predictive variable of pAF in males. Several potential mechanisms can account for the association between increased AF burden and BNP levels. BNP is secreted predominantly from ventricular myocytes, and a small amount of BNP release from the atrium occurs in patients with AF as a response to atrial stretch. Elevated BNP levels in AF patients may also reflect increased left atrial pressure and stretch, being independent of the ventricular secretion of BNP. Therefore, increased mechanical atrial stretch itself promotes the secretion of BNP, and BNP might predict both the frequency and progression of AF [16, 17]. This reflects a mechanism by which increased left atrial pressure of AF in men is different from that in women.

Serum bilirubin, which is the catabolic product of the heme catabolic pathway, has long been used as a biomarker for hepatic metabolic and excretory capacity. Experimental evidence has shown that bilirubin might act as a powerful antioxidant and anti-inflammatory agent in biological functions and is associated with different cardiovascular diseases [18]. In patients with coronary artery disease, bilirubin levels have an inverse relationship with cardiovascular events [19]. In contrast, the bilirubin level has been positively correlated with heart failure and pulmonary hypertension in clinical observation studies [20, 21]. The bilirubin level in AF patients is unclear. One clinical study found that higher serum bilirubin levels were associated with AF recurrence in paroxysmal AF patients following catheter ablation [22]. We came to similar results, in which Tbil and Ibil were higher in the pAF group. In addition, we also observed that Ibil was an independent predictive factor of pAF in females. In patients with pAF, bilirubin, as an anti-inflammatory and antioxidant substance, may be compulsorily increased.

Anemia is known to be associated with poor prognosis in cardiovascular diseases. Relative hypochromia of erythrocytes, defined as a reduced MCHC, is a surrogate of iron deficiency [23]. Hammadah et al. [24] indicated that a lower MCHC is an independent predictor of increased mortality risk in nonanemic patients with HF. Kleber et al. [25] also reported that MCHC is a common and strong independent predictor of increased mortality in acute HF after adjusting for anemia. Nevertheless, there has been no research on the association between MCHC and AF until now. In the present study, patients with pAF had a larger MCHC than the SR group, and a higher MCHC was an independent predictive factor of pAF. The reason may be that patients with pAF have intermittent episodes of arrhythmia and transient abnormal heart function, which leads to a corresponding hypoxia-induced haemoglobin increase.

This study has limitations. First, this was a cross-sectional study, and there was no patient follow-up; therefore, these results may be prone to selection or information bias. Second, this was a single-center study, and the sample size was small; thus, it is not known whether these findings are generalizable, and thus, they need to be further confirmed in the future. Third, the biomarkers of inflammatory and oxidative stress were limited, and the characteristics were evaluated at only one time point.

## 5. Conclusion

In pAF patients, age, smoking, and MCHC are independent predictive factors of pAF. BNP is an independent predictive biomarker of pAF in males; age and Ibil are independent predictive factors of the occurrence of pAF in females.

## Figures and Tables

**Figure 1:** Differences in the levels of sST2, TIMP-1, BNP, Ibil, MCHC, and LA in pAF and non-AF. The levels of ST2, TIMP-1, BNP, Ibil, and MCHC were significantly higher and the LA diameter was significantly larger in the pAF group than in the non-AF group. ST2: suppression of tumorigenicity 2; pAF: proximal atrial fibrillation.

**Table 1:** Baseline clinical characteristics of the participants stratified according to pAF status.

Characteristic	All (*n* = 181), *n* (%)	pAF (*n* = 68), *n* (%)	Non-AF (*n* = 113), *n* (%)	*P* value
Age, years	52.9 ± 15.1	60.4 ± 9.9	48.3 ± 15.9	<0.0001
CAD	6 (3.3)	1 (1.5)	5 (4.4)	0.517
HTN	64 (35.4)	35 (51.5)	29 (22.1)	0.007
DM	22 (12.2)	9 (13.2)	13 (11.5)	0.73
HF	7 (3.9)	3 (4.4)	4 (3.5)	0.918
Smoking	36 (19.9)	27 (39.7)	9 (8.0)	<0.0001
Drinking	4 (2.2)	0 (0)	4 (3.5)	0.741
Diuretic	3 (1.7)	0 (0)	3 (2.7)	0.687
Statin	20 (11.0)	16 (23.5)	4 (3.5)	0.067
ACEI/ARB	16 (8.8)	7 (10.3)	9 (8.0)	0.523
CCB	8 (4.4)	0 (0)	8 (7.1)	0.984
Beta-blockers	7 (3.9)	1 (1.5)	6 (5.3)	0.497

CHA2DS2-VASc score				
0 or 1, *n* (%)	125	42	83	0.231
2 or 3, *n* (%)	44	18	26	
≥4, *n* (%)	12	8	4	
Mean score	1.32	1.53	1.19	

HAS-BLED score				
≥3, *n* (%)	9 (5)	7 (10.3)	2 (1.77)	0.001
Mean score	0.63	0.94	0.45	
LA (mm)	37.22 ± 7.77	39 ± 7.25	35.62 ± 7.92	0.01
LVEF (%)	61.56 ± 10.88	60.22 ± 11.82	62.78 ± 9.85	0.165
LVEDD (mm)	46.77 ± 7.35	46.35 ± 7.27	47.14 ± 7.45	0.534
LVESD (mm)	30.34 ± 6.18	30.68 ± 5.53	30.04 ± 6.7	0.546

CAD: coronary artery disease; HTN: hypertension; DM: diabetes mellitus; HF: heart failure; ACEI: angiotensin-converting enzyme inhibitors; ARB: angiotensin receptor blocker; CCB: calcium channel blocker; LA: left atrium diameter; LVEF: left ventricular ejection fraction; LVEDD: left ventricular end-diastolic dimension; LVESD: left ventricular end-systolic dimension.

**Table 2:** Baseline laboratory examination of the participants stratified according to pAF status.

Characteristic	All (*n* = 181), *n* (%)	pAF (*n* = 68), *n* (%)	Non-AF (*n* = 113), *n* (%)	*P* value
RBC (10^9^/l)	4.72 ± 0.45	4.75 ± 0.44	4.71 ± 0.45	0.605
WBC (10^9^/l)	6.62 ± 1.61	6.45 ± 1.45	6.73 ± 1.7	0.258
PLT (10^12^/l)	232.33 ± 60.18	212 ± 46	244 ± 64	<0.0001
Hb (g/l)	146.35 ± 15.41	150 ± 15	144 ± 15	0.005
CREA (*μ*mol/l)	66.56 ± 16.46	72.4 ± 17.3	63 ± 14.9	<0.0001
UA (*μ*mol/l)	331.38 ± 86.66	348.23 ± 80.21	321 ± 89.3	0.42
GLU (mmol/l)	5.66 ± 1.81	5.72 ± 1.46	5.62 ± 2.0	0.714
GA (%)	14.13 ± 2.45	14.4 ± 2.4	14.0 ± 2.5	0.323
HCY (*μ*mol/l)	14.25 ± 8.59	14.4 ± 7	14.1 ± 9.5	0.814
TIMP-1 (ng/ml)	74.04 ± 22.11	82.01 ± 25.05	69.24 ± 18.67	<0.0001
sST2 (pg/ml)	11.22 ± 4.92	12.76 ± 4.73	10.3 ± 4.82	<0.0001
BNP (pg/ml)	76.06 (21.5–109.75)	102.7 (48.5–151)	54.04 (13–79)	<0.0001
ALT (U/l)	25.08 ± 19.32	25.04 ± 21.07	25.1 ± 18.23	0.986
AST (U/l)	23.55 ± 13.37	24.56 ± 21.07	22.95 ± 7.47	0.434
TP (g/l)	72.69 ± 5.75	70.40 ± 5.64	74.08 ± 5.38	<0.0001
Alb (g/l)	45.66 ± 4.54	43.80 ± 4.43	46.78 ± 4.24	<0.0001
Glo (g/l)	27.03 ± 4.56	26.59 ± 5.51	27.29 ± 3.88	0.318
Tbil (*μ*mol/l)	9.54 ± 4.83	14.95 ± 6.23	11.67 ± 5.15	<0.0001
Dbil (*μ*mol/l)	3.38 ± 1.74	3.42 ± 1.92	3.35 ± 1.62	0.79
Ibil (*μ*mol/l)	9.55 ± 3.83	11.52 ± 4.09	8.31 ± 3.22	<0.0001
LDH (U/l)	183.73 ± 47.86	176.60 ± 49.9	188.18 ± 46.21	0.118
TG (mmol/l)	1.67 ± 1.11	1.80 ± 1.15	1.59 ± 1.07	0.216
Tcho (mmol/l)	4.76 ± 1.03	4.77 ± 1.07	4.76 ± 1.01	0.923
LDL-c (mmol/l)	2.9 ± 0.88	2.95 ± 0.93	2.86 ± 0.85	0.518
HDL-c (mmol/l)	1.25 ± 0.31	1.15 ± 0.25	1.31 ± 0.33	<0.0001
LP(a) (mmol/l)	0.16 (0.03–0.17)	0.154 (0.03–0.17)	0.166 (0.04–0.17)	0.746
FFA (mmol/l)	0.53 (0.36–0.7)	0.522 (0.36–0.67)	0.537 (0.34–0.73)	0.715
C1q (mg/l)	175.19 ± 33.29	174.69 ± 30.71	177.28 ± 35.16	0.633
hs-CRP (mg/l)	2.01 ± 3.19	2.44 ± 4.17	1.74 ± 2.37	0.214
D-dimer (ng/ml)	95.41 ± 78.03	94.76 ± 83.9	95.80 ± 74.65	0.932
FDP (ug/ml)	0.46 (0.1–0.7)	0.437 (0–0.6)	0.479 (0.1–0.7)	0.59
FIB (g/l)	3.09 (2.5–3.4)	3.404 (2.53–3.48)	2.895 (2.5–3.3)	0.107
HCT (%)	42.25 ± 3.88	42.866 ± 3.720	41.878 ± 3.948	0.097
MCV (fl)	88.96 ± 6.29	90.12 ± 5.68	88.27 ± 6.56	0.054
MCH (pg)	31.15 ± 2.87	31.72 ± 1.62	30.80 ± 3.36	0.035
MCHC (g/l)	346.32 ± 12.15	350.43 ± 11.43	343.85 ± 12.42	<0.0001
RDW-SD (fl)	42.47 ± 3.73	42.70 ± 2.64	42.33 ± 4.26	0.527
RDW-CV (%)	13.1 ± 1.24	12.99 ± 0.60	13.17 ± 1.49	0.347
MPV (fl)	10.72 ± 0.99	10.78 ± 0.96	10.69 ± 1.00	0.567
PCT (%)	0.25 ± 0.06	0.23 ± 0.05	0.26 ± 0.07	0.432
PDW (%)	13.42 ± 2.26	13.23 ± 2.40	13.54 ± 2.18	0.374

WBC: white blood cell; RBC: red blood cell; PLT: platelet count; Hb: haemoglobin; UA: uric acid; CREA: creatinine; Glu: fasting blood glucose; GA: glycated albumin; HCY: homocysteine; TIMP-1: tissue inhibitors of metalloproteinase-1; sST2: soluble suppression of tumorigenicity-2; BNP: B-type natriuretic peptide; ALT: alanine aminotransferase; AST: aspartate transaminase; TP: total protein; Alb: albumin; Glo: globulin; Tbil: total bilirubin; Dbil: direct bilirubin; Ibil: indirect bilirubin; LDH: lactate dehydrogenase; TG: triacylglycerol; Tcho: total cholesterol; LDL-c: low-density lipoprotein cholesterol; HDL-c: high-density lipoprotein cholesterol; LP(a): lipoprotein (a); FFA: free fatty acid; C1q: anti-complement 1q antibody; hs-CRP: high-sensitivity C-reactive protein; FDP: fibrinogen degradation products; FIB: fibrinogen; HCT: haematocrit; MCV: mean red blood cell volume; MCH: mean corpuscular haemoglobin; MCHC: mean corpuscular haemoglobin concentration; RDW-SD: red blood cell distribution width-standard deviation; RDW-CV: red blood cell distribution width-cell volume; MPV: mean platelet volume; PCT: platelet haematocrit; PDW: platelet distribution width.

**Table 3:** Multivariable logistic regression analysis of factors associated with pAF.

Factor	OR	OR 95% CI	*P* value
Age	1.075	1.035–1.118	<0.0001
Smoking	4.538	1.559–13.205	0.006
MCHC	1.062	1.019–1.106	0.004

**Table 4:** Differences in clinical characteristics between males and females with pAF.

Characteristic	All (*n* = 68), *n* (%)	Males (*n* = 46), *n* (%)	Females (*n* = 22), *n* (%)	*P* value
Smoking	27 (39.7)	25 (54.3)	2 (9.1)	<0.0001
Age, years	60.63 ± 9.94	59.76 ± 9.5	62.45 ± 10.81	0.229
HTN	35 (51.5)	23 (50)	12 (54.5)	0.728
WBC (10^9^/l)	6.44 ± 1.45	6.46 ± 1.45	6.43 ± 1.48	0.946
PLT (10^12^/l)	212.28 ± 46.47	202.80 ± 45.91	232.09 ± 42.02	0.014
Hb (g/l)	150.44 ± 15.42	156.67 ± 12.62	137.41 ± 12.42	<0.0001
CREA (*μ*mol/l)	72.44 ± 17.28	77.55 ± 17.29	61.78 ± 11.64	<0.0001
UA (*μ*mol/l)	348.58 ± 79.66	321.50 ± 70.13	361.30 ± 82.3	0.045
TIMP-1 (ng/ml)	82 ± 25.06	86.31 ± 26.64	72.0 ± 18.87	0.039
ST2 (pg/ml)	12.76 ± 4.73	13.40 ± 4.87	11.43 ± 4.23	0.109
BNP (pg/ml)	113.34 (48.75–155.5)	108.68 (40.5–141.5)	124.58 (56.5–192.5)	0.777
TP (g/l)	70.4 ± 5.64	70.55 ± 5.00	70.06 ± 6.90	0.768
Alb (g/l)	43.8 ± 4.43	44.02 ± 4.83	43.35 ± 3.51	0.569
Tbil (*μ*mol/l)	14.95 ± 6.23	16.27 ± 6.66	12.19 ± 4.11	0.01
Ibil (*μ*mol/l)	11.53 ± 5.1	12.40 ± 5.52	9.71 ± 3.51	0.041
HDL-c (mmol/l)	1.15 ± 0.25	1.10 ± 0.23	1.24 ± 0.25	0.024
MCH (pg)	31.72 ± 1.62	32.13 ± 1.13	30.87 ± 2.12	0.002
MCHC (g/l)	350.43 ± 11.44	353.52 ± 10.71	343.95 ± 10.33	0.001
LA (mm)	39 ± 7.25	38.98 ± 4.93	39.05 ± 10.63	0.972

HAS-BLED score				
≥3, *n* (%)	7 (10.3)	4 (8.7)	3 (13.6)	
Mean score	0.94	0.88	1.05	0.382

WBC: white blood cell; RBC: red blood cell; PLT: platelet count; Hb: haemoglobin; UA: uric acid; CREA: creatinine; TIMP-1: tissue inhibitors of metalloproteinase-1; ST2: soluble suppression of tumorigenicity-2; BNP: B-type natriuretic peptide; TP: total protein; Alb: albumin; Tbil: total bilirubin; Ibil: indirect bilirubin; HDL-c: high-density lipoprotein cholesterol; MCH: mean corpuscular haemoglobin; MCHC: mean corpuscular haemoglobin concentration; LA: left atrium.

**Table 5:** Multivariable logistic regression analysis of factors associated with pAF in males and females.

	Factor	OR	OR 95% CI	*P*-value
Females	Age	1.107	1.016–1.206	0.02
	Ibil	2.303	1.158–4.582	0.017

Males	BNP	1.015	1.002–1.029	0.029

## Data Availability

The datasets used and analyzed during the current study are available from the corresponding author on reasonable request.
